# Tooth CT Image Segmentation Method Based on the U-Net Network and Attention Module

**DOI:** 10.1155/2022/3289663

**Published:** 2022-08-19

**Authors:** Sha Tao, Zhenfeng Wang

**Affiliations:** School of Electrical Engineering, Tongling University, Tongling 244000, China

## Abstract

Traditional image segmentation methods often encounter problems of low segmentation accuracy and being time-consuming when processing complex tooth Computed Tomography (CT) images. This paper proposes an improved segmentation method for tooth CT images. Firstly, the U-Net network is used to construct a tooth image segmentation model. A large number of feature maps in downsampling are supplemented to downsampling to reduce information loss. At the same time, the problem of inaccurate image segmentation and positioning is solved. Then, the attention module is introduced into the U-Net network to increase the weight of important information and improve the accuracy of network segmentation. Among them, subregion average pooling is used instead of global average pooling to obtain spatial features. Finally, the U-Net network combined with the improved attention module is used to realize the segmentation of tooth CT images. And based on the image collection provided by West China Hospital for experimental demonstration, compared with other algorithms, our method has better segmentation performance and efficiency. The contours of the teeth obtained are clearer, which is helpful to assist the doctor in the diagnosis.

## 1. Introduction

In recent years, deep learning has developed rapidly and has been applied to many fields of image processing [1]. Among them, image segmentation is one of the key topics in modern computer vision research [2]. The effect of image segmentation in the medical field is getting more and more attention. Whether it is pathological analysis, diagnosis and treatment, or clinical surgical navigation, image segmentation can play a better auxiliary treatment effect. It can quickly identify the lesion and reduce the cost of medical care [3]. Traditional image segmentation is done manually layer by layer by experienced doctors, which takes a long time. The segmentation results of these regions of interest (RoI) are quite different among different doctors [4]. The automatic segmentation of CT images can significantly reduce the workload of doctors and improve the accuracy and consistency of RoI segmentation [5]. At present, modern medical CT mainly includes multiple spiral CT and cone beam CT (CBCT). CBCT is more commonly used in dentistry, which has the characteristics of short scanning time and low radiation dose [6]. Because the bones of the teeth are closely intertwined with some soft tissues, the CT scan image of the tooth will become very blurred. And there are differences in the grayscale value distribution between teeth. There may also be differences in the grayscale value of the same tooth, the topological structure is more complicated, and it is not easy to distinguish [7]. Therefore, accurate and efficient medical image segmentation algorithms are necessary.

Image segmentation currently does not have a unified general-purpose algorithm. Most algorithms are aimed at specific types of objects, looking for their characteristic points to construct specific energy functions to achieve segmentation [8, 9]. In medical CT image segmentation, the traditional template-based segmentation method has gradually become one of the common methods of RoI delineation in radiotherapy [10]. Kaur et al. [11] proposed a CT image segmentation technique based on a mixture of spatial intuitionistic fuzzy *C*-means clustering and spatial regularization level set methods. It can integrate the details of the spatial image and accurately and effectively extract the kidney disease image in the CT image. Li et al. [12] proposed a new validity index after evaluating the tightness and separation of the dataset twice. The effectiveness of the proposed metrics is verified using a large number of synthetic datasets and some typical CT images. This metric is suitable for datasets with arbitrarily shaped clusters that are susceptible to noise corruption. It is beneficial to cluster analysis and computer-aided detection systems. Shi et al. [13] proposed an improved potential well function combined with a level set model for tooth segmentation. The segmentation speed and accuracy are improved. Ji et al. [14] proposed a level set method for tooth shape extraction from head CBCT images, which achieved high accuracy.

However, due to the frequent changes in the anatomy of human organs, it is difficult for traditional methods to establish a universal template based on fixed images. Moreover, even the same RoI may have large differences due to differences in patient size and age [15]. In recent years, deep learning methods have been widely used. For example, stacked autoencoder, deep belief networks (DBN), recurrent neural network (RNN), and convolutional neural network (CNN) have been extensively studied in related fields [16, 17]. Sun [18] proposed the Darknet-53 network for extracting tooth image features and multiscale prediction. The SE module is added to the network to improve the network performance. Li et al. [19] proposed a CNN-based stereo image segmentation framework. The use of coherent parallax propagation solves the inevitable inaccuracy problem of the parallax calculated from the stereo image pair. Then, the pixels propagated through the coherent parallax and the high-confidence pixels of the target probability map generated by the CNN architecture will be used to generate the initial reliable pixels to perform the segmentation based on the energy minimization framework. CNN automatically extracts multilevel visual features by learning a large number of mapping relationships between inputs and outputs [20]. Zhou et al. [21] proposed a three-level network based on 3D U-Net to segment a single tooth. But the relationship between alveolar bone and teeth is very important when orthodontists make orthodontic plans for patients. Kadry et al. [22] used the pretrained VGG-UNet system to extract ISL fragments from brain MRI slice test images and extract COVID-19 infection from lung CT images. Tong et al. [23] propose an extended version of U-Net, which uses the concept of triple attention mechanism to segment skin lesions. The segmentation results are more accurate for complex skin lesions such as shape, size, color, and texture. But the algorithm is more complicated and time-consuming. Zhang et al. [24] proposed a triple crossover U-Nets (TIU-Nets) for glioma segmentation. The proposed TIU-Nets are composed of binary class segmentation U-Net (BU-Net) and multiclass segmentation U-Net (MU-Net) and have achieved better performance. Tooth CT images are relatively simple for skin lesion images and brain MRI images. Miki et al. [25] studied the application of CNN to classify tooth types on dental CT images, which is beneficial to obtain high classification accuracy without the need for accurate tooth segmentation. Chung et al. [26] proposed a neural network for per-pixel labeling to segment frames using instances that are robust to metal artifacts.

Compared with CNN, U-Net adds upsampling and downsampling processes, generates images of different resolutions, and convolves images of various resolutions [27]. To this end, a tooth CT image segmentation method using the U-Net network is proposed. For this paper, the main contributions are as follows:

1. Since the segmentation effect of fully convolutional networks (FCN) is relatively rough, the proposed method uses the U-Net network for image segmentation. And through data enhancement, a more ideal tooth CT image segmentation result can be obtained
2. In order to improve the segmentation speed of the network and reduce the loss of precision, the attention module is integrated in the U-Net network and improved. The Subregional Average Pooling (SAP) module is used to obtain the initial channel weight information, and the CE module is used to expand the low-level channel attention

This paper is divided into four sections in total.  Section 1 introduces the research significance and technical difficulties of topic selection and classifies the existing image semantic segmentation methods. On this basis, summarize the innovative points of the proposed method.  Section 2 elaborates on the proposed method, using the U-Net network combined with the improved attention module to segment the tooth CT image.  Section 3 discusses the experimental results and uses relevant standards to evaluate the performance of the proposed method.  Section 4 is the conclusion.

## 2. Materials and Methods

### 2.1. U-Net

U-Net is a U-Net network structure proposed by Olaf Ronneberger in 2015. It is a semantic segmentation network based on FCN, which matches the form of downsampling during the upsampling process to keep it consistent [28, 29]. On this basis, a large number of feature maps in the downsampling stage are added to the downsampling to fill in the information lost during the operation. Because its structure is symmetrical like U-shaped, it is named the U-Net network.

U-Net has special advantages in processing medical images. In solving the problem of the lack of sample images in medical images, elastic deformation is used to complete data enhancement [30]. Elastic deformation is a relatively common type of deformation in actual cells, so it is very suitable for medical image processing [31]. The algorithm of data enhancement is used to make the neural network model learn the invariance of elastic deformation. In the case of a small dataset, the network has good elastic deformation adaptability. The segmentation can be completed correctly when meeting the elastic deformation of the medical image [32]. The U-Net network has excellent effect on cell segmentation, and its segmentation effect is shown in Figure 1.

The U-Net network has attracted attention from the medical field since its inception. On the basis of U-Net, many scholars have improved this structure. For example, Milletari's 3D deformation structure V-Net and Drozdzal's changes to the skip structure have added many variants to the U-Net network.

### 2.2. Attention Module

In order to increase the weight of effective features and improve the accuracy of segmentation, we have added an attention mechanism module to the network [33]. The human visual attention mechanism is divided into data-driven and task-driven [34]. This paper uses a data-driven attention mechanism module. The level of attention weight is positively correlated with the importance of the corresponding location information. The input unit with high weight has a decisive effect on the output result. Firstly, global average pooling (GAP) is performed on each channel to obtain the vector of 1 × 1 × *K*. More than two fully convolutional (FC) layer transformations are done. Sigmoid and ReLU activation functions are used. The extraction network is shown in Figure 2.

In the attention module, first use GAP to shrink the data output from the downsampling layer from *W* × *H* × *K* to 1 × 1 × *K*, which is expressed as follows:

(1) $$\begin{array}{c} z_{c}=f_{\text{sq}}\left(u_{c}\right)\frac{1}{H\times W}\overset{H}{\underset{i=1}{\sum }}\overset{W}{\underset{j=1}{\sum }}u_{c}\left(i,j\right), \end{array}$$

where *f*_sq_ represents the GAP function.

After that, the network performs two FC operations. *C* represents the dimensionality reduction coefficient, which can be adjusted according to the specific network. The best performance is obtained when *C* = 16 is demonstrated experimentally; the formula is as follows:

(2) $$\begin{array}{c} \begin{array}{c} s_{c}=f_{\text{ex}}\left(z_{c},W\right)=\varepsilon \left(g\left(z_{c},W\right)\right)=\varepsilon \left(W_{2}\delta \left(W_{1}z_{c}\right)\right),\\ W_{1},W_{2}\in R^{\left(K/C\right)\times K}, \end{array} \end{array}$$

where *ε* and *δ* represent sigmoid and ReLU activation functions, respectively. *f*_ex_ is the FC function.

Then, perform the scale operation. Based on the number of channels unchanged, the data is changed to *W* × *H* × *K*; the calculation is as follows:

(3) $$\begin{array}{c} X_{c}=f_{\text{scale}}\left(u_{c},s_{c}\right)=s_{c}\cdot u_{c}, \end{array}$$

where *f*_scale_ is the scale operation function.

Before the network joins the attention module, for an input image with a batch of 256 and a size of 224 × 224, a forward propagation takes 42 ms. After adding the attention module, it takes 47 ms. After reducing the complexity, there is still time to increase, but it can be ignored compared with the improvement of segmentation accuracy [35].

Because segmentation task scenes are often complex and changeable, using GAP is too simple. The features needed for segmentation cannot be extracted effectively [36]. In response to this problem, the SAP structure was proposed. The structures of GAP and SAP are shown in Figure 3.

As shown in Figure 3, GAP turns a channel feature with a dimension of *H* × *W* × *K* into a feature with the size of 1 × 1 × *K*. In SAP, a feature with a size of *H* × *W* × *K* is transformed into a new feature with a size of *m* × *n* × *k*, so that some spatial information is retained. Then, through a convolution kernel of size *m* × *n*, the obtained feature map is transformed into a feature of size *H* × *W* × *K*. The feature extraction network with the attention module is shown in Figure 4.

First increase the number of channels and use a 1 × 1 convolution. Because 1 × 1 convolutional layers are usually used to adjust the number of channels between network layers and control the model complexity, it enables interaction and information integration across channels. At the same time, the nonlinear characteristics can be greatly increased while keeping the size of the feature map unchanged, making the network very deep. Then, add the high-level and low-level channel attention weights. Finally, multiply the new weights with higher-order features [37, 38]. The size range of the updated weight is (0, 2), which can not only reduce but also expand the feature value [39].

The obtained channel feature $\hat{F}$ connects a 1 × 1 convolution *φ*_*r*_ and sigmoid activation function *ε*, *r* ∈ [1, *K*]. The output *ε*_SAP_ of the SAP module is

(4) $$\begin{array}{c} \begin{array}{c} \varepsilon_{\text{SAP}}=\left[\varepsilon_{1},\varepsilon_{2},\cdots ,\varepsilon_{r},\cdots ,\varepsilon_{K}\right],\\ \varepsilon_{r}=\varepsilon \left(\overset{K}{\underset{i=1}{\sum }}\varphi_{r}*{\hat{F}}_{i}\right). \end{array} \end{array}$$

Finally, define the high-order attention distribution obtained by the SAP module as . The low-level attention distribution after passing the CE module is *ε*_*l*_(·). Then, it can be used for the updated attention distribution *ε*_*F*_:

(5) $$\begin{array}{c} \varepsilon_{F}=\varepsilon_{l}\left(\cdot \right)+\varepsilon_{h}\left(\cdot \right). \end{array}$$

The recalibrated characteristic map $\hat{U}$ can be obtained as

(6) $$\begin{array}{c} \hat{U}=U\varepsilon_{F}. \end{array}$$

### 2.3. Network Structure

The attention module is integrated into the U-Net network to obtain a network model for tooth CT image segmentation. The structure is shown in Figure 5.

Using 3 layers of 3 × 3 convolutional layers, change the ordinary 3 × 3 convolution to dilated convolution with expansion rate 2, and the resolution of the output feature map is 1/16 of the input. Atrous spatial pyramid pooling (ASPP) is used to provide multiscale information in the U-Net network. That is, on the basis of spatial pyramid pooling, a hole convolution with different expansion rates is added, and global information is added through SAP and image features. The features output by ASPP are upsampled, added to a low-level feature that has undergone a 3 × 3 convolution, and then merged with a 3 × 3 convolution. Finally, it is upsampled and restored to the original image size [40].

## 3. Results and Discussion

The experiment is based on the Keras framework, which is developed by Google. It uses TensorFlow and Theano packages to integrate many basic neural network structures and some mature algorithms. The experimental dataset used is dental CT data provided by West China Hospital. The operating system is Windows 10, the CPU is an 8 GB Intel Core i7-6700, and the GPU is NVIDIA Ge Force GTX 1070.

When training, the optimization method uses random gradient descent (SGD). Its momentum parameter is set to 0.9, and the weight decay rate is 1 × 10^−4^. The learning rate uses the initial learning rate learning rate = 8 × 10^−3^ multiplied by (1 − current_iter/max_iter)^power^ to reduce the strategy. Where power = 0.9, current_iter is the current number of iterations, and max_iter is the maximum number of iterations in the training process. The number of experimental training iterations is 800.

### 3.1. Data Preprocessing

Based on the segmentation task of the U-Net network, the final output is closely related to the quality of the input image. In view of the fact that some of the tooth CT images have similar grayscale value, shapes, or textures, image enhancement methods are used to preprocess the input image data to improve image contrast. Histogram equalization (HE) is a basic method of image enhancement. And adaptive histogram equalization (AHE) is improved through HE. AHE improves local contrast, enhances the edge sharpness of each area of the image, and improves the shape, texture, and boundary information of the teeth. Before entering the network, the normalized image grayscale value is (0,1), and the image size is 512 × 512.

In order to overcome the overfitting phenomenon of neural networks, the proposed method adopts enhancement techniques such as random cropping, flipping, grayscale perturbation, and shape perturbation on the data image to overcome this problem. The gray level disturbance in the training set can improve the stability of the network, thereby improving the performance of the prediction set network.

The CT image and contour image are deformed by affine transformation to form shape disturbance. In the deformation, the coordinates of the 3 vertices (upper left, upper right, and lower left) are first obtained. Then, each point moves randomly, and the range of random movement is the image length. Finally, affine transformation is performed on the entire image.

After image enhancement, the training set (400 images) and the validation set (100 images) are both enlarged 3 times. A total of 1500 image data were obtained for experimental training and parameter adjustment.

### 3.2. Evaluation Index

In the experiment, mean pixel accuracy (MPA) and mean intersection over union (MIoU) are used as indicators to evaluate the performance of the proposed method.

Assume that *n*_*ii*_ represents the number of correct segmentation. *n*_*ij*_ represents the number of pixels that originally belonged to class *i* but were divided into class *j*. *n*_*ji*_ represents the number of pixels that originally belonged to class *j* but were divided into class *i*. There are *k* + 1 categories (including *k* classes and an empty class or background class).

MPA calculates the proportion of pixels that are correctly segmented in each class and then finds the average of all classes. The calculation is as follows:

(7) $$\begin{array}{c} \text{MPA}=\frac{1}{k+1}\overset{k}{\underset{i=0}{\sum }}\frac{n_{ii}}{\sum_{j=0}^{k}n_{ij}}. \end{array}$$

MIoU calculates the ratio of intersection and union of two sets. Calculate the pixel intersection ratio within each pixel category, and then, calculate the average:

(8) $$\begin{array}{c} \text{MIOU}=\frac{1}{k+1}\overset{k}{\underset{i=0}{\sum }}\frac{n_{ii}}{\sum_{j=0}^{k}n_{ij}+\sum_{j=0}^{k}n_{ji}-n_{ii}}. \end{array}$$

Due to its strong representativeness, high efficiency, and simplicity, MIoU has become the current general image segmentation evaluation index. Therefore, MIoU is used as the main evaluation index of the experiment.

### 3.3. Comparison of the Proposed Algorithms

According to the proposed method, the final tooth CT image segmentation result is obtained. The segmentation comparison result of the proposed method and the traditional U-Net network is shown in Figure 6.

It can be seen from Figure 6 that the proposed method can segment the tooth CT image more effectively than the traditional U-Net network. The effect of tooth edge extraction is significantly better than that of U-Net. However, affected by some noise, there is a certain shadow in the center of the segmented image. Therefore, the performance of the U-Net network before and after the improvement is quantitatively analyzed. The results of MPA and MIoU and the time to complete the segmentation are shown in Table 1.

As can be seen from Table 1, the proposed method improves the U-Net network by using the attention mechanism. MPA is 85.91%, and MIoU is 83.73%, which is superior to the U-Net network in terms of segmentation accuracy. However, due to the complexity of the segmentation model, the time to complete the segmentation has also increased. Compared with the U-Net network, the time has increased by 28 ms. However, from an overall point of view, the proposed method still has a large application advantage in tooth CT image segmentation.

In order to further demonstrate the performance of the proposed method, compare it with References [13, 18] and [21]. The segmentation results of tooth CT images obtained by each method are shown in Figure 7.

It can be seen from Figure 7 that the tooth profile obtained by the proposed method is clearer and is closest to the original image.  Figure 7(b) adopts the traditional segmentation method combined with the level set model [13], the segmentation effect is not good, and the contour is blurred. Figures 7(c) and 7 (d) use learning algorithms for segmentation [18, 21], but a single algorithm needs to be improved in processing complex tooth images. Therefore, the effectiveness of the proposed method for segmentation of tooth CT images can be demonstrated.

The quantitative analysis results of different methods are shown in Table 2.

It can be seen from Table 2 that the segmentation performance of the proposed method is the best, with MPA of 85.91% and MIoU of 83.73%. It completes the detection speed of 126 ms, but the model is more complicated than that of Reference [13], so the time is slightly longer. The traditional method used in Reference [13] has low segmentation accuracy for complex teeth CT images, with MIoU of only 68.05%. But it takes the shortest time to complete the detection, which is 74 ms. Reference [18] chooses the Darknet-53 network for extracting tooth image features and multiscale prediction. Overall, it has good segmentation performance, but the algorithm is not effective in learning complex features, and the segmentation accuracy needs to be improved. Reference [21] segmented teeth based on a three-level network of 3D U-Net. But the model is more complicated, so it takes a long time, 183 ms. From a comprehensive point of view, the proposed method has obvious application advantages in tooth CT image segmentation.

## 4. Conclusions

With the development of today's society, medical standards have put forward higher requirements in people's lives. There are many representative computational intelligence algorithms, such as monarch butterfly optimization (MBO) [41], earthworm optimization algorithm (EWA) [42], elephant herding optimization (EHO) [43], and moth search (MS) algorithm [44, 45]. With the continuous increase in the number of CT images and MRI images, the segmentation of medical images by manpower alone can no longer meet the demand. Therefore, the use of deep learning for automatic segmentation has attracted wide attention from scholars. We propose a tooth CT image segmentation method using the U-Net network. The attention module is integrated into the U-Net network, and the SAP and CE modules are used to improve the performance of the network. Based on the tooth CT image dataset provided by West China Hospital, the improved network was demonstrated experimentally. With comprehensive comparison, the method in this paper has better segmentation performance and segmentation efficiency. The contours of the teeth obtained are clearer, which is helpful to assist the doctor in the diagnosis. The proposed method only performs segmentation for tooth images and has not been used for segmentation of other medical images. In the following research, the proposed method will be applied to other organizations to improve the generalization ability of the proposed method. And in-depth pruning of the network is carried out to improve network efficiency.

## Figures and Tables

**Figure 1:** U-Net network segmentation cell diagram.

**Figure 2:** Feature extraction network with the attention module.

**Figure 3:** Structure comparison between GAP and SAP.

**Figure 4:** Feature extraction network with the attention module.

**Figure 5:** U-Net network structure combined with the improved attention module.

**Figure 6:** Comparison of segmentation results before and after the improvement of the U-Net network.

**Figure 7:** Segmentation results of different methods.

**Table 1:** Comparison of segmentation performance before and after the improvement of the U-Net network.

Methods	MPA (%)	MIoU (%)	Execution time (ms)
U-Net	82.37	80.19	98
Improved U-Net	85.91	83.73	126

**Table 2:** Comparison of segmentation performance of different methods.

Methods	MPA (%)	MIoU (%)	Execution time (ms)
Ref. [13]	69.11	68.05	74
Ref. [18]	80.03	79.24	167
Ref. [21]	84.76	83.19	183
The proposed method	85.91	83.73	126

## Data Availability

The data included in this paper are available without any restriction.
